The article "Artesunate Suppresses the Growth of Lung Cancer Cells by Downregulating the AKT/Survivin Signaling Pathway" was retracted in 2023. Reasons: signs of a paper mill; compromised peer review; unreliable results or conclusions.

# Artesunate Suppresses the Growth of Lung Cancer Cells by Downregulating the AKT/Survivin Signaling Pathway

**DOI:** 10.1155/2022/9170053

**Published:** 2022-03-25

**Authors:** Weiwei Zhang, Ning Ning, Jie Huang

**Affiliations:** ^1^Department of traditional Chinese Medicine, Hunan Provincial People's Hospital, Changsha 410005, Hunan, China; ^2^Scientific Research Office of Hunan Provincial People's Hospital, Changsha, Hunan 410005, China; ^3^Department of Emergency, Hunan Provincial People's Hospital, Changsha, Hunan 410005, China

## Abstract

NSCLC (non-small-cell lung cancer) is the deadliest cancer in the world. Artesunate is one of the most potent and rapidly acting antimalarial agents. Recently, emerging evidence has suggested the anticancer function of artesunate. In our work, we aimed to investigate the molecular mechanism of artesunate-induced growth inhibition in human lung adenocarcinoma cells and reported that the anticancer effects of artesunate is related to its ability in downregulating AKT/Survivin signaling in A549 cells. The effect of artesunate on the proliferation of A549 cells was determined by CCK-8 assay and colony formation assay; its effect on A549 cell apoptosis was evaluated by lactate dehydrogenase (LDH) release assay. The role of artesunate on the activation of AKT/Survivin signaling was analyzed by western blot and quantitative QPCR. Finally, we used two mouse tumor models to investigate the function of artesunate on the *in vivo* growth of lung cancer cells. Artesunate treatment caused significant growth inhibition and apoptosis in A549 cells. Mechanistically, artesunate downregulated the activation of AKT/Survivin signaling. In agreement, hyperactivation of AKT signaling restored artesunate-induced growth inhibition in A549 cells. In mouse lung cancer models, artesunate administration significantly reduced the growth of A549 cells and LLC cells in nude mice and immunocompetent mice, respectively. Our findings suggest that artesunate serves as a potential tumor suppressor in lung cancer and hopefully can provide new insight into the development of therapeutic strategies in the clinical lung cancer treatment.

## 1. Introduction

Artemisinin is a sesquiterpene lactone extracted from Artemisia annua, which is a semisynthetic derivative of artemisinin. Artesunate is a class of antimalarial drug that controls the symptoms of malaria, but its modulatory roles in tumor growth and the underlying molecular mechanisms remain relatively poorly understood. Artemisinin and its derivatives have been included in the anticancer drug screening and anticancer activity research program by the National Cancer Institute (NCI) in the United States due to their proven anticancer effects [1]. Lung cancer accounts for the top cancer death worldwide. According to all lung cancer data, non-small-cell lung cancer (NSCLC) accounts for over 80% of lung cancer, with high invasion and metastasis rate. Most patients die from metastasis and recurrence. According to the report, artesunate could lead the apoptosis of human hepatoma cells in vitro, with no obvious effect on expression [2]. However, it is extremely important to furtherly study the influence of artesunate on the growth of lung cancer cells.

AKT, also known as protein kinase B, is a serine/threonine kinase with a 70% homology between its kinase domain and protein kinases A and C [3]. AKT signaling has great effects on signal regulation during tumor formation and is involved in tumor cell proliferation, apoptosis inhibition, mesenchymal neovascularization, and tumor cell invasion and metastasis [4]. As a well-characterized downstream target effector of AKT signaling, Survivin is one of significant family members in inhibitors of apoptosis. Survivin is expressed during embryonic development, but its expression was low in adult tissues after development. In many transformed cell lines and tumor tissues, Survivin expression was reported to be enhanced [5]. Survivin plays an important oncogenic role in ovarian cancer, laryngeal cancer, breast cancer, and cholangiocarcinoma and serves an important prognostic indicator [6]. Furthermore, Survivin was reported to be correlated with tumor metastasis in oral cancer, gastric cancer, prostate cancer, and lung cancer [7]. An earlier study has reported that artesunate induced cell apoptosis via a Bak- and AIF-mediated caspase-independent intrinsic pathway, in which BH-3 only protein Bim, as a key initiator, played an important role in activating the Bak signaling [8]. In the current study, CCK8 results showed that artesunate significantly decreased the proliferation of A549 cells in a concentration-dependent manner. The colony formation assay also showed that artesunate inhibited the colony formation ability of A549 cells. Survivin can be deregulated in cancer by several mechanisms, such as amplification of the Survivin locus on chromosome 17q25(15), demethylation of Survivin exons [9], increased promoter activity [10], and the upstream signaling in the PI3K/AKT or MAPK pathways [11].

In this study, we found that artemisinin serves as a tumor suppressor in lung cancer. Artemisinin administration not only inhibited the growth of A549 lung cancer cells *in vitro* but also delayed *in vivo* growth in nude mice and immune-competent mice. The effect of artemisinin was attributed to its ability in downregulating the activation of AKT/Survivin signaling pathway.

## 2. Materials and Methods

### 2.1. Reagents

Artesunate and dimethyl sulfoxide (DMSO) were made a purchase from Sigma (USA). Antibodies of p-AKT, AKT, Survivin, c-caspase-3, and *β*-actin were all obtained from Proteintech.

### 2.2. Cell Culture

A549 cells (ATCC® CCL-185) and Lewis lung carcinoma (LLC, ATCC® CRL-1642) cells were obtained from American Type Culture Collection (ATCC). Cells were cultured in DMEM and supplemented with 10% FBS, 20 mM HEPES, 100 U/ml penicillin, and 100 mg/ml streptomycin. Cells were maintained in a humidified, 95% CO_2_ atmosphere at 37°C.

### 2.3. CCK-8 Assay

We used Cell Counting Kit-8 (Dojindo Laboratories, Kumamoto, Japan) to analyze the cell viability according to the description by Li and Altieri [10]. In brief, after treatment with different concentrations of artesunate for 24 h, the cells were incubated with 10 *μ*l of CCK-8 solution at 37°C for another 1 h. Then, the medium was abandoned and DMSO was used to dissolve the formation of formazan crystals. A microplate spectrophotometer is to measure the absorbance. The calculations of cell viability were based on previous study.

### 2.4. Lactate Dehydrogenase (LDH) Release Assay

Within 24 hours, different concentrations of artesunate treat A549 cells. The cell culture supernatant was collected, and the levels of LDH were evaluated using the LDH Assay Kit (Beyotime, Shanghai, China) based on the instructions of thr manufacturer. The measurement of OD values was on a Promega™ Microplate Reader (Promega, Madison, WI, USA).

### 2.5. Colony Formation Assay

The colony formation assay measured the cytotoxic effects of artesunate. Briefly, A549 cells were seeded onto 6-well plates (2000 cells/well). After incubation overnight, artesunate deal with the cells with different concentrations within 24 hours. After that, cells with complete medium were breezed for another following 10 days.

PBS washed the colonies forming on plates, then being fixed in methanol, and lastly being stained with 1% methylrosanilinium chloride. A microscope (Olympus, Japan) was used to count the colonies and to measure the colony's percentage in each treatment group.

### 2.6. Quantitative Real-Time Polymerase Chain Reaction (qQPCR)

To synthesize first-strand cDNA with a synthesis kit of iScript cDNA (Bio-Rad, Hercules, CA, USA) depending on manufacturer's directions, the analyses of real-time qPCR were performed using a QPCR mixture containing 1 *μ*M of each primer and EvaGreen Supermix (Bio-Rad).

A StepOnePlus real-time QPCR system (Applied Biosystems, Foster City, CA, USA) was used to perform amplifications at 95°C for 15 s and at 60°C for 30 s. Each sample was examined in triplicate, and glyceraldehyde phosphate-3 dehydrogenase mRNA level was regarded as an inner control. Primer sequences are illustrated as follows: GAPDH: forward 5′-GTCTCCTCTGACTTCAACAGCG, reverse 5′-ACCACCCTGTTGCTGTAGCCAA; Bcl2: GAPDH: forward 5′ATCGCCCTGTGGATGACTGAGT, reverse 5′GCCAGGAGAAATCAAACAGA GG; Bax: GAPDH: forward 5′TCAGGATGCGTCCACCAAGAAG, reverse 5′-TGTGTCCACGGCGGCAATCATC; and Survivin: GAPDH: forward 5′CCACTGAGAACGAGCCAGACTT, reverse 5′-GTATTACAGGCGTAAGCCACCG.

## 3. Statistics Analysis

The illustration of all results adopted the mean ± SD according to the independent experiments unless without indication. Through the tests of Student *T* and Spearman's rank correlation and one-way ANOVA of Dunnett, we find that there are big and obvious differences among the groups. All statistical analyses were performed with the Statistical Program for Social Sciences (SPSS), version 17.0.

### 3.1. Western Blots

60 mm plates were used to seed A549 cells, and artesunate was used after overnight incubation to treat artesunate. Then, RIPA (Beyotime, Shanghai, China), containing protease inhibitor cocktail, was used to lyse the cells. The lysate was centrifuged at 15,000 rpm for 15~20 min at 4°C. The BCA protein assay kit (Beyotime, Shanghai, China) was used to detect the concentration of proteins. The samples of protein were subjected to electrophoresis, and then, they were transferred to the poly-vinylidene difluoride transfer membranes (Millipore, Billerica, MA). The blots were blocked with 5% nonfat milk for 1 h at room temperature and incubated with primary antibody at 4°C. Then, the blots were incubated with horseradish peroxidase-conjugated secondary antibodies for 1 hour. An ECL kit was used with the immunoreactive bands. The software of ImageJ was used to analyze the immunoreactive band density.

### 3.2. Mouse Tumor Models

6 ~ 8-week athymic nude mice (*n* = 6/group) or C57BL/6 mice (*n* = 7/group) were purchased from Shanghai Laboratory Animal Center (Shanghai, China). 8 × 10^5^ A549 or LLC cells were injected subcutaneously into the left flank of mice. One week after tumor inoculation, mice were intratumoral injected with artesunate (80 mg/kg) or the same volume of PBS every 3 days. Tumor volume was monitored with a caliper and then calculated using the formula: *V* = Length × (Width)2/2. Fifteen to twenty days postinoculation, when tumor volume reached approximately 1500 mm^3^, mice were used for cervical dislocation in the following experiments.

## 4. Results

### 4.1. Artesunate Effectively Inhibits the Viability and Proliferation of A549 Cells

First, CCK8 assay was used to investigate the influence of artesunate on A549 cell proliferation. As presented in Figure 1(a), artesunate treatment magnificently stopped the growth of A549 cells in a manner with dose dependency. We further evaluated the antiproliferative effects of artesunate using the colony formation assay. As shown in Figure 1(b), being compared to untreated cells, we found that artesunate significantly inhibited colony formation capacity of A549 cells in a manner with dose dependency. Moreover, in the controlled group, the artesunate-treated cells colonies were much smaller. Next, we evaluated the role of artesunate on the apoptosis of A549 cells by LDH release assay. The results showed that artesunate treatment dose dependently induced A549 cell apoptosis (Figure 1(c)). Collectively, our results suggest that artesunate stopped the viability and proliferation of A549 cells.

### 4.2. Artesunate Inhibited the Activation of AKT/Survivin Signaling Pathway

The PI3K/AKT pathway mediates the effects of extracellular signals on various cellular processes, such as cell growth, proliferation, survival, and death. Previous research has reported that restraint of PI3K/AKT signaling induced apoptosis of A549 lung cancer cells [12]. We found that artesunate effectively suppressed the phosphorylation level of AKT in A549 cells in a dose-dependent manner (Figure 2(a)). Comparing with controlled cells after the treatment of 24 hours, there was a decreasing phenomenon, such as percentage of phosphorylated AKTSer473 was reduced to 26.2% (25 *μ*g/ml), 53.5% (50 *μ*g/ml), and 48.8% (100 *μ*g/ml) separately (Figure 2(a)). Next, we determined whether artesunate could inhibit the expression of Survivin. As illustrated in Figure 2(b), exposure of A549 cells to artesunate at concentrations of 25, 50, and 100 *μ*M/ml for 24 h expressively reduced the protein level of Survivin in a dose-dependent manner in comparison with controlling A549 cells. Moreover, artesunate treatment significantly enhanced the grade of cleaved caspase-3 in A549 cells (Figure 2(c)). Taken together, artesunate causes improvement of inhibition and apoptosis of A549 cells by suppressing AKT/Survivin signaling.

### 4.3. Activation of the AKT Protected A549 Cells from Artesunate-Induced Growth Inhibition

Based on the above findings, we then investigated whether the restoration of AKT activation could reverse the antiproliferative effects of artesunate on A549 cells. Cells were preincubated for 1 h in the presence or absence of SC97 and then treated with artesunate. In Figure 3(a), MTT assay was used to detect the cell viability.

In Figure 3(b), the colony formation assay was performed to detect proliferation, and the representative histogram for colony formation in A549 cells. In Figure 3(c), the relative mRNA expressions of AKT, c-caspase-3, Survivin, Bax, and Bcl2 were analyzed by RT-QPCR. In Figure 3(d), the protein levels of p-AKT, AKT, Survivin, and c-caspase-3 were analyzed by western blot. The band densities were quantified by Eagle Eye II software; ^∗^*P* < 0.05, ^∗∗^*P* < 0.01, and ^∗∗∗^*P* < 0.001.

Eventually, A549 cells were pretreated with DMSO or SC79 for 24 h followed by artesunate (50 ng/ml) treatment for another 24 h. As shown in Figure 3(a), SC79 massively enhanced cell proliferation compared with untreated or DMSO-treated A549 cells. The effect of SC79 on cell proliferation was furtherly proved by the colony formation assay (Figure 3(b)). As expected, SC97 treatment significantly raised the level of p-AKT and Survivin, while reducing the level of cleaved-caspase-3 (Figure 3(c)). In addition, SC97 treatment resulted in a significantly downregulated expression of proapoptotic protein Bax but upregulated the expression of antiapoptotic protein Bcl2 (Figure 3(d)). The results suggest that artesunate exerts its antiproliferative role by downregulated AKT activation.

### 4.4. Artesunate Suppresses Tumor Growth in Nude Mice and Immune-Competent Mice

Next, we examined if artesunate could suppress the in vivo growth of lung cancer cells. We further examined the effect of artesunate on tumor growth in immune-competent mice. Lewis lung carcinoma (LLC) cells were subcutaneously inoculated into C57BL/6 mice. Similar to its effect on A549 tumors, artesunate administration significantly inhibited LLC growth in mice (Figures 4(a) and 4(b)). Likely, tumor levels of Survivin and Bcl2 were downregulated by artesunate (Figures 4(c) and 4(e)) and were positively correlated with the weight of LLC tumors (Figures 4(d) and 4(f)).

To this end, A549 cells were inoculated subcutaneously into nude mice, which were then subjected to artesunate gavage. The results presented that artesunate meaningfully inhibited the growth of A549 cells in mice, as evidenced by the reduced tumor volume and tumor weight (Figures 5(a) and 5(b)). Furthermore, artesunate significantly downregulated the expression of Survivin and Bcl2 in tumor tissues as assessed by RT-QPCR (Figures 5(c) and 5(e)). Importantly, there was a positive correlation between the grade of Survivin or Bcl2 in tumor tissues and tumor weight in artesunate-administered mice (Figures 5(d) and 5(f)), suggesting that the efficiency of artesunate to suppress tumor growth was correlated with its effort to downregulate Survivin expression. Collectively, artesunate exerts the antitumor function both in vitro and in vivo.

## 5. Discussion

Previous evidence has implicated that artemisinin and its derivative artesunate can be used as potential anticancer agents [12, 13]. In our work, we aimed to investigate the mechanism of artesunate-induced growth inhibition in lung adenocarcinoma cells of human, which reported that the anticancer effects of artesunate is related to its ability in downregulating AKT/Survivin signaling in A549 cells. Thus, the inhibition effect of artesunate on cell proliferation can be used as an anticancer drug in clinic in patients with lung cancer, especially in those with hyperactivation of AKT.

An earlier study has reported that artesunate induced cell apoptosis by a Bak/AIF-mediated caspase-independent internal signal, in which BH-3/Bim played an active role in activating the Bak pathway [8]. In this study, CCK8 data showed artesunate obviously decreased the proliferation of A549 cells via a concentration-dependent way. On the other hand, artesunate significantly inhibited the clonogenesis of A549 cells. In addition, we also observed a dose-dependent cytotoxic effect of artesunate against lung cancer cells. Importantly, the antitumor function of artesunate was further substantiated using two mouse lung cancer models.

Cell proliferation inhibition is a significant toxic effect through which some anticancer drugs decrease the viability of cancer cells. Therefore, it is crucial to examine whether inhibition cell proliferation caused by anticancer drugs is involved in inhibition of antiapoptotic gene expression, such as Survivin, which is associated with malignant cell proliferation, progression, and chemotherapy resistance [14–17]. In our study, our data showed artesunate-induced proliferation inhibition of A549 cells was associated with activation exogenous caspase signaling. Accumulating studies show Survivin could regulate cell apoptosis by inhibiting caspase-3/7 activity. Caspase-3 is the functional executor of the caspase family, which is mainly involved in apoptosis and plays a key role in the cleavage of PARP. It has been known that the decreased expression of Survivin results in increased caspase-3 activity and cleavage of PARP. In cancer, Survivin can be degraded by a variety of mechanisms, such as amplification of Survivin sites on chromosome 17q25 [18], demethylation of Survivin exons [9], increased promoter activity [10], and upstream activation of PI3K/AKT or MAPK signaling pathways [11].

The AKT signaling pathway is an effective oncogenic regulator, widely involved in tumor cell growth, invasion, migration, and survival, which is frequently low expressed in human tumors such as non-small-cell lung cancer (NSCLC) and head and neck squamous cell carcinoma (HNSCC). The effect of artesunate on phosphorylation of AKT has also been reported in endothelial cells in vitro [19]. There is evidence to suggest that the AKT-mediated survival pathway may inhibit apoptosis by stimulating Survivin synthesis in various cancer cell lines [20–22].

However, the role of AKT pathway in artesunate-induced apoptosis is unclear. In the present study, the results suggest that AKT may be involved in artesunate-induced cell proliferation inhibition. On the other hand, artesunate could significantly decrease the phosphorylation of AKT in a concentration-dependent manner, while the total levels of AKT showed no change. Meanwhile, we enhanced the AKT pathway in artesunate therapy in SC97 cells, a chemical agonist that increases AKT activity, to determine if there is a mechanism of inhibited cell proliferation by artesunate.

## 6. Conclusion

We found that low nontoxic concentrations of SC97 significantly alleviated the effect of artesunate and rescued the cell proliferation inhibition. Further, pretreatment with SC97 partially inhibited changes in Survivin and the caspase-3 activity. These results clearly indicate the involvement of AKT pathway activation in artesunate-mediated cell proliferation inhibition. In conclusion, artesunate can induce the growth inhibition and apoptosis in lung cancer cells via dampening AKT/Survivin, indicating its potential role in the clinical treatment of lung cancer.

## Figures and Tables

**Figure 1:** Influences of artesunate on the viability of A549 cells. (a) A549 cells were treated with 0, 25, 50, and 100 *μ*g/ml artesunate for 24 h. Then, the cell viability was determined by MTT assay. (b) A549 cells were treated with the different concentrations of artesunate for 24. The performance of colony formation assay to detect proliferation, and the typical histogram in colony formation of A549 cells. (c) Cell apoptosis was evaluated by LDH release assay. The expression of the data was used with the mean ± SD based on the results from three separate experiments. Mean ± SD expressed data, and then, Dunnett's test one-way ANOVA analyzed the data. ^∗^*P* < 0.05, ^∗∗^*P* < 0.01, and ^∗∗∗^*P* < 0.001.

**Figure 2:** Artesunate inhibits the AKT/Survivin signaling pathway. (a) A549 cells were greeted with the referential concentrations of artesunate for 1 day; Survivin, Bax, and Bcl2 were analyzed by QPCR. (b) A549 cells were treated with the indicated concentrations of artesunate for 1 day; Survivin, p-AKT, and c-caspase-3 were analyzed by RT-QPCR. (c) A549 cells were treated with the indicated concentrations of artesunate for 24 h; p-AKT, AKT, Survivin, and c-caspase-3 proteins were analyzed by western blot. The band densities were quantified using Eagle Eye II software. Data were expressed as mean ± SD from three independent experiments and analyzed by one-way ANOVA followed by Dunnett's test. ^∗^*P* < 0.05, ^∗∗^*P* < 0.01, and ^∗∗∗^*P* < 0.001.

**Figure 3:** AKT agonist protected A549 cells from artesunate-induced growth inhibition.

**Figure 4:** Artesunate inhibits the growth of LLC cells in immunocompetent mice. 8 × 10^5^ LLC cells were subcutaneously inoculated into nude mice. (a) Tumor growth were monitored. (b) Tumor weight was measured at day 19. (c, e) The expression of Survivin and Bcl2 was evaluated by RT-QPCR. (d, f) The correlation between Survivin or Bcl2 expression and tumor weight was analyzed by Spearman's rank correlation test. ^∗^*P* < 0.05, ^∗∗^*P* < 0.01, and ^∗∗∗^*P* < 0.001.

**Figure 5:** Artesunate restraints the development of A549 cells in nude mice. 8 × 10^5^ A549 cells were subcutaneously inoculated into naked mice. (a) Tumor growth were monitored. (b) Tumor weight was measured at day 20. (c, e) The expression of Survivin and Bcl2 was evaluated by RT-QPCR. (d, f) The correlation between Survivin or Bcl2 expression and tumor weight was analyzed by Spearman's rank correlation test. ^∗^*P* < 0.05, ^∗∗^*P* < 0.01, and ^∗∗∗^*P* < 0.001.

## Data Availability

The datasets used and/or analyzed during the current study are available from the corresponding author on reasonable request.
